The article "Effect of Calcification Based on Computer-Aided System on CT-Fractional Flow Reserve in Diagnosis of Coronary Artery Lesion" was retracted in 2023. Reasons: signs of a paper mill; compromised peer review; unreliable results or conclusions.

# Effect of Calcification Based on Computer-Aided System on CT-Fractional Flow Reserve in Diagnosis of Coronary Artery Lesion

**DOI:** 10.1155/2022/7020209

**Published:** 2022-01-17

**Authors:** Dongliang Fu, Xiang Xiao, Tong Gao, Lina Feng, Chunliang Wang, Peng Yang, Xianlun Li

**Affiliations:** ^1^Department of Cardiology, Integrated Traditional Chinese and Western Medicine, China-Japan Friendship Hospital, No. 2 East Yinghua Road, Chaoyang District, Beijing 100029, China; ^2^Graduate School, Peking Union Medical College, Beijing 100730, China; ^3^Beijing Escope Tech Co., Ltd., Beijing, China

## Abstract

This study was to analyze the diagnostic value of coronary computed tomography angiography (CCTA) and fractional flow reserve (FFR) based on computer-aided diagnosis (CAD) system for coronary lesions and the possible impact of calcification. 80 patients who underwent CCTA and FFR examination in hospital were selected as the subjects. The FFR value of 0.8 was used as the dividing line and divided into the ischemic group (FFR ≤ 0.8) and nonischemic group (FFR > 0.8). The basic data and imaging characteristics of patients were analyzed. The maximum diameter stenosis rate (MDS %), maximum area stenosis rate (MAS %), and napkin ring sign (NRS) in the ischemic group were significantly lower than those in the nonischemic group (*P* < 0.05). Remodeling index (RI) and eccentric index (EI) compared with the nonischemic group had no significant difference (*P* > 0.05). The total plaque volume (TPV), total plaque burden (TPB), calcified plaque volume (CPV), lipid plaque volume (LPV), and lipid plaque burden (LPB) in the ischemic group were significantly different from those in the non-ischemic group (*P* < 0.05). MAS % had the largest area under curve (AUC) for the diagnosis of coronary myocardial ischemia (0.74), followed by MDS % (0.69) and LPV (0.68). CT-FFR had high diagnostic sensitivity, specificity, accuracy, truncation value, and AUC area data for patients in the ischemic group and nonischemic group. The diagnostic sensitivity, specificity, accuracy, cutoff value, and AUC area data of CT-FFR were higher in the ischemic group (89.93%, 92.07%, 95.84%, 60.51%, 0.932) and nonischemic group (93.75%, 90.88%, 96.24%, 58.22%, 0.944), but there were no significant differences between the two groups (*P* > 0.05). In summary, CT-FFR based on CAD system has high accuracy in evaluating myocardial ischemia caused by coronary artery stenosis, and within a certain range of calcification scores, calcification does not affect the diagnostic accuracy of CT-FFR.

## 1. Introduction

Cardiovascular disease, also known as circulatory system disease, is a series of diseases involving the circulatory system. It has become the primary noncommunicable disease threatening global public health. The World Health Organization (WHO) global noncommunicable status report predicts that by 2030, the number of deaths from cardiovascular diseases will reach 22.2 million every year [1, 2]. Coronary heart disease is a heart disease caused by atherosclerotic lesions in the coronary artery, resulting in stenosis or obstruction of the vascular cavity, myocardial ischemia, hypoxia, or necrosis [3]. It has been proposed that the pathophysiological basis of acute coronary syndrome is the rupture of “vulnerable” single criminal plaque, which promotes the formation of acute thrombosis in situ and leads to the occurrence of acute coronary events [4, 5]. In short, the fight against cardiovascular disease has become a common challenge for all mankind regardless of region, race, and country.

There are many imaging diagnosis methods for cardiovascular diseases, mainly including X-ray, echocardiography, angiocardiography, MRI, and CT. X-ray chest film can display the size, shape, position, and contour of cardiac large vessels and observe the relationship between the heart and adjacent organs, but its imaging parts overlap, it is difficult to distinguish details, and it does not have three-dimensional imaging characteristics; so, it is impossible to directly provide hemodynamic data [6, 7]. Echocardiography can not only make anatomical diagnosis of cardiovascular diseases but also make functional diagnosis. It can observe the intracardiac movement, ventricular wall thickness, and the connection of cardiac great vessels from any angle, but it is seriously affected by factors such as sound, visual field, resolution, and operator experience [8–10]. Although MRI has high temporal resolution and soft tissue resolution, it has poor effect on coronary artery imaging due to the thin diameter of coronary artery, tortuous shape, and more adipose tissue in adjacent parts [11, 12]. CT can measure the human body with highly sensitive instruments according to the different X-ray absorption and transmittance of different human tissues and show the small lesions in any part of the body [13]. Coronary computed tomography angiography (CCTA) has become an important method for early diagnosis of coronary heart disease as a rapid noninvasive imaging method developed in the past decade. The increasing number of CCTA examinations and related medical research and applications urgently requires automatic segmentation of coronary arteries in CCTA images. This can not only provide rich postprocessing tools for clinical diagnosis but also improve the efficiency of clinical diagnosis. It can also provide quantitative evaluation indicators for the diagnosis of coronary heart disease and improve the accuracy and automation of diagnosis. This study proposes an automatic coronary artery segmentation algorithm, which can accurately segment the coronary artery lumen area according to the structure and image characteristics of the vascular lumen and surrounding tissues. However, it can only provide the stenosis degree and wall information of coronary artery lumen and cannot accurately determine whether stenosis leads to distal hemodynamic abnormalities resulting in myocardial ischemia.

Although the image diagnosis method is more and more accepted by doctors, the traditional image diagnosis can only be qualitative observation, without quantitative information, cannot realize the conversion from data to information, and largely depends on the experience and ability of doctors, which is greatly limited. Computer aided diagnosis (CAD) system combines computer technology with image processing to analyze the patient's image information, finally detect the lesion, and help clinicians obtain more accurate evaluation results [14, 15]. CAD system can avoid the influence of doctors' subjective feelings and improve different diagnostic outcomes caused by doctors' personal experience and knowledge differences, which plays an important role in promoting the radiological diagnosis of clinical medicine [16]. At present, the measurement of fractional flow reserve (FFR) combined with performing invasive coronary angiography is the gold standard for the diagnosis of hemodynamic abnormalities caused by coronary artery stenosis [17, 18]. CT-FFR is based on computational fluid dynamics and uses CCTA data to calculate FFR value. It is a new noninvasive method to measure the hemodynamic abnormalities of stenotic coronary artery.

The use of CT-FFR in the diagnosis of coronary artery disease is the focus of current research. Therefore, 80 patients with coronary artery disease were studied. The basic data and imaging characteristics of the patients were analyzed, and the diagnostic value of CT-FFR based on CAD system for coronary artery disease was comprehensively evaluated.

## 2. Materials and Methods

### 2.1. Research Objects

In this study, 80 patients with confirmed coronary artery disease by imaging examination, aged 35-80 years, who were admitted to hospital for CCTA examination and FFR examination from May 2, 2019 to June 5, 2021, were selected as the study subjects. 49 males and 31 females were divided into 40 cases of the coronary ischemia group (FFR ≤ 0.8) and 40 cases of the noncoronary ischemia group (FFR > 0.8). This study has been approved by the ethics committee of hospital, and the family members of the patients are informed of this study and sign informed consent.

Inclusion criteria are as follows: (1) patients of voluntary cooperation examination, (2) patients who signed informed consent, and (3) patients' image quality was good.

Exclusion criteria are as follows: (1) patients had a fluctuation range of invasive FFR value, (2) patients had abnormal origin of coronary artery, (3) patients had a history of coronary stent implantation, and (4) patients received coronary artery bypass grafting.

### 2.2. CCTA Examination

The patients were examined by CCTA using the second-generation ostentatious dual-source CT instrument of Siemens, Germany. Patients were given breath-holding training before scanning to reduce image respiratory motion artifacts and sublingual nitroglycerin 3 minutes before scanning to expand the coronary artery. The ECG activity of patients was monitored throughout the whole process. If the heart rate of patients exceeded 70 times per minute, about 60 mg esmolol hydrochloride injection was intravenously injected. At a speed of 5.2 mL/s, 60 mL of nonionic contrast agent of iopamidol and 50 mL of 0.9% sodium chloride injection were intravenously injected before elbow. The contrast agent tracer method was used to select the region of interest at the aortic root to monitor the CT attenuation value. When the CT attenuation value reached 100HU, it was waited for 5 seconds to start scanning. The scanning range was from 1 cm above aortic arch to 1 cm below cardiac diaphragm. Scanning parameters are as follows: detector collimation 1.5 × 125 × 0.5 mm. The thickness is 0.65 mm. The tube current is 350 mAs/turn. Rotation time is 0.3 seconds/cycle, and tube voltage is120 kV.

### 2.3. FFR Test

FFR is defined as the ratio of the maximum blood flow that can be obtained in the myocardial region supplied by this vessel to the maximum blood flow that can be obtained theoretically under normal conditions in the same region in the presence of stenotic lesions in the coronary arteries, that is, the ratio of the mean intracoronary pressure at the distal end of the stenosis (Pd) to the mean aortic pressure (Pa) at the coronary artery orifice under the maximum myocardial hyperemia. Coronary angiography was performed by Judkins method through femoral artery puncture. FFR was measured with a pressure/temperature guide wire of 0.036 mm in diameter. Adenosine triphosphate was injected into the median elbow vein at a flow rate of about 150 *μ*g/kg to induce coronary circulation load. The theoretical normal value of FFR is “1,” if FFR0.8 lesion does not induce myocardial ischemia.

### 2.4. Automatic Coronary Artery Segmentation Algorithm

The tubular structure similarity is applied to the vascular enhancement of medical images. Firstly, the tubular structure similarity function is set as follows.

(1) $$\begin{array}{c} S\left(i,j,h;\alpha \right)=0\;\beta_{1}>0\text{or}\beta_{2}>0,\\ S\left(i,j,h;\alpha \right)=\begin{array}{cc} \left[1-\exp\left(-\frac{{E_{A}}^{2}}{2a^{2}}\right)\right]\left[1-\exp\left(-\frac{{E_{B}}^{2}}{2b^{2}}\right)\right]\left[1-\exp\left(-\frac{W^{2}}{2c^{2}}\right)\right] & \text{others} \end{array}. \end{array}$$

*β*_1_, *β*_2_, and *β*_3_ are the eigenvalues of Hessian matrix. *E*_*A*_ and *E*_*B*_ are used for the characteristic differences between different forms such as disc-shaped and spot-shaped structures, *E*_*A*_ = |*β*_1_|/|*β*_2_| and $E_{B}=\left|\beta_{3}\right|/\sqrt{\beta_{1}\beta_{2}}$. *W* represents the brightness difference between the label and the surrounding background, $W=\sqrt{{\beta_{1}}^{2}+{\beta_{2}}^{2}+{\beta_{3}}^{2}}$. *a* is the proportion factor of influencing *E*_*A*_, *b* is the proportion factor of influencing *E*_*B*_, and *c* is the proportion factor of influencing *W*, 0 < *S*(*i*, *j*, *h*; *α*) < 1.

In general, the radius of the coronary artery is between 2 and 7 mm, and not all pixels can meet the current eigenvalues under single-scale conditions; so, the similarity function needs to be calculated under multiscale conditions.

(2) $$\begin{array}{c} S\left(i,j,h;\alpha \right)=\underset{\alpha_{\min}\leq \alpha \leq \alpha_{\max}}{\max}\left\{\alpha^{\kappa }S\left(i,j,h;\alpha \right)\right\}. \end{array}$$

*κ* is the regularization coefficient. In practice, it is found that the above algorithm still has the problems of low computational efficiency and inaccurate seed point extraction in single scale. Therefore, this study uses the position information of the ascending aorta to automatically locate the region of interest, so as to reduce the range of seed point search area and reduce the computational complexity. In addition, the three-dimensional geometric properties of coronary pixels and the brightness difference between coronary artery, bone tissue, and pulmonary vascular background are used to restrict the extraction of coronary seed points and improve the accuracy of seed points. The final segmentation algorithm flow is shown in Figure 1.

### 2.5. CAD System of Coronary Artery

Coronary artery CAD system is a large unit of clinical medical image. In order to improve the effectiveness and reliability of clinical aided diagnosis, this study designs a customizable and easy to expand coronary artery CAD system (Figure 2). The system mainly includes data layer, model layer, and implementation layer. The data layer can realize the interaction and access of coronary CTA volume data, input the collected coronary data into the coronary CAD system for processing, and save the diagnosis results for clinical communication. The model layer contains the core technologies and algorithms of CAD, which can extract valuable information from massive and complex data. The implementation layer is a platform for mutual communication between the system and doctors. It can intuitively, quickly, and concisely display the data processing results to users according to a certain workflow, such as visual display of segmentation results, data query information list, and operation log.

In this study, the function of the whole system is divided into multiple models for design, including command module, digital imaging, and communications in medicine (DICOM) module, eXtensible Markup Language (XML) log module, report module, image module, script module, data processing module, and algorithm module. The command module can uniformly process the input information in the process of clinical diagnosis and coordinate the data transmission between functional modules. DICOM module can analyze and process different kinds of DICOM files to ensure the correctness of the results and provide extended functions through the script system. The XML log module can parse and record the execution of each command, accurately locate the program exceptions, and output the parameter information during execution. The report module can automatically generate the corresponding graphic report according to the operation in the process of clinical diagnosis. The image module can provide the function of drawing various regions of interest. The script module can customize and expand the function of coronary artery CAD using Python language. The data processing module can provide the functions of saving, managing, and querying various data in the whole detection process. The algorithm module is an embedded coronary artery CAD algorithm (Figure 3).

### 2.6. Clinical Data

Clinical information of patients was collected through the medical record system, including demographic characteristics (age, height, sex, weight), clinical history (lipidemia, hypertension, diabetes, smoking history), and biochemical examination results (total cholesterol (TC), high-density lipoprotein cholesterol (HDL-C), low density lipoprotein cholesterol (LDL-C), triglyceride (TG), and fasting plasma glucose (FPG)).

### 2.7. Image Features

Maximum diameter stenosis rate (MDS %) and maximum area stenosis rate (MAS %) are measured and calculated, MDS% = (Blood vessel diameter‐Diameter of lumen at narrowest position/Blood vessel diameter) × 100%, and MAS% = (Cross sectional area of blood vessel‐Cross‐sectional area of blood vessel at narrowest point/Cross sectional area of blood vessel) × 100% . The total plaque volume (TPV), total plaque burden (TPB), calcified plaque volume (CPV), calcified plaque burden (CPB), noncalcified plaque volume (NCPV), noncalcified plaque burden (NCPB), lipid plaque volume (LPV), lipid plaque burden (LPB), fiber plaque volume (FPV), and fiber plaque burden (FPB) were measured. Napkin-ring sign (NRS), remodeling index (RI), and eccentricity index (EI) were calculated.

### 2.8. Statistical Methods

The data of this study were analyzed by SPSS19.0 statistical software. The measurement data were expressed by mean ± standard deviation ($\overset{¯}{x\pm s}$), and the counting data were expressed by percentage (%). Single factor analysis of variance was used for pairwise comparison. The difference was statistically significant (*P* < 0.05).

## 3. Results

### 3.1. Comparison of Basic Data of Patients

As shown in Table 1, the age, height, weight, male ratio, hyperlipidemia, hypertension, diabetes, smoking history, total cholesterol, HDL-C, LDL-C, triglycerides, and FPG of the ischemic group and the nonischemic group were not statistically significant (*P* > 0.05).

### 3.2. Imaging Data

Figure 4 shows the signs of normal coronary artery. The tube wall is smooth, and there is no stenosis in the lumen.  Figure 5 shows the image of coronary artery calcification without stenosis. There is limited severe calcification near the heart, and the pipe wall is not smooth, but there is no obvious stenosis at the location of calcification.  Figure 6 shows diffuse calcification with stenosis in the proximal segment of the left coronary artery, with severe stenosis in the corresponding segment.

### 3.3. Comparison of CCTA Indexes between the Two Groups

The MDS %, MAS %, and NRS of patients in the ischemic group were significantly lower than those in the nonischemic group (*P* < 0.05) (Figure 7). There was no significant difference in RI and EI between the ischemic group and nonischemic group (*P* > 0.05).

There was significant difference in TPV, TPB, CPV, LPV, and LPB between the ischemic group and the nonischemic group (*P* < 0.05) (Figure 8). There was no significant difference in CPB, NCPV, NCPB, FPV, and FPB between the ischemic group and nonischemic group (*P* > 0.05).

### 3.4. Diagnostic Performance of Quantitative Indexes for Coronary Myocardial Ischemia

From Figures 9 and 10, the diagnostic AUC area of MAS % is the largest (0.74), followed by MDS % (0.69), and LPV (0.68).

### 3.5. Diagnostic Performance of CT-FFR in Two Groups of Patients

From Table 2, the diagnostic sensitivity, specificity, accuracy, cut-off value, and AUC area of CT-FFR for patients in the ischemic group and nonischemic group are high, but the comparison between them is not statistically significant (*P* > 0.05).

## 4. Discussion

In recent years, cardiovascular disease has developed into one of the diseases that seriously threaten human health, and its early diagnosis and intervention are particularly important [19]. As a noninvasive imaging technology commonly used in clinic, CCTA has been proved to have high accuracy in diagnosing coronary artery diameter stenosis of cardiovascular diseases. With the development of CT imaging technology, the spatial resolution, temporal resolution, and density resolution of CCTA have been greatly improved, and CCTA has complete evaluation ability for lesions with lumen diameter of more than 1.5 mm [20]. In this study, 80 patients who underwent CCTA examination and FFR examination in the hospital were selected as the research objects. With FFR value of 0.8 as the dividing line, they were divided into the ischemic group (FFR ≤ 0.8) and nonischemic group (FFR > 0.8). The basic data showed that there were no significant differences in age, height, weight, male ratio, hyperlipidemia, hypertension, diabetes, smoking history, total cholesterol, HDL-C, LDL-C, triglycerides, and FPG between the ischemic group and nonischemic group (*P* > 0.05), which provided reliability for subsequent research results. Comparing the degree of lumen stenosis and the characteristic indexes of vulnerable plaque, it is found that the MDS %, MAS %, and NRS in the ischemic group are significantly lower than those in the nonischemic group (*P* < 0.05), while there is no significant difference in RI and EI compared with the nonischemic group (*P* > 0.05), which is similar to the research results of Zhang et al. (2020) [21], indicating that there are great differences in the degree of lumen stenosis between ischemic and nonischemic patients. In addition, it was also found that there were significant differences in TPV, TPB, CPV, LPV, and LPB between the ischemic group and the nonischemic group (*P* < 0.05), indicating that there were differences in the characteristics of vulnerable plaques between the ischemic and nonischemic patients. In conclusion, the characteristics of coronary artery disease (coronary lumen area stenosis or vulnerable plaque component index, etc.) may have better diagnostic value for coronary disease-specific myocardial ischemia.

The diagnostic performance of quantitative indexes for coronary myocardial ischemia was analyzed. The results showed that the diagnostic AUC area of MAS % was the largest (0.74), followed by MDS % (0.69) and LPV (0.68), which was consistent with the research results of Ghanem et al. (2019) [22], indicating that MAS % was better than MDS % in the diagnosis of coronary lesion specific myocardial ischemia. This may be because MAS % can provide more lumen information. On the one hand, because complex lesions such as diffuse lesions and bifurcation lesions are common, MDS % can only provide diameter stenosis information at the narrowest lumen, while MAS % can provide stenosis area of lumen cross section at the narrowest lumen to reflect lumen stenosis more truly. On the other hand, in the presence of eccentric plaque, MDS % often overestimates the true degree of stenosis of the lumen due to the evaluation of the diameter stenosis at the most severe stenosis [23, 24]. By analyzing the diagnostic performance of CT-FFR in the two groups, it was found that the diagnostic sensitivity, specificity, accuracy, cut-off value, and AUC area of CT-FFR in the ischemic group and nonischemic group were high, but the comparison between them was not statistically significant (*P* > 0.05). This shows that CT-FFR based on computer-aided diagnosis system has high accuracy in evaluating myocardial ischemia caused by coronary artery stenosis, and calcification does not affect the diagnostic accuracy of CT-FFR within a certain calcification score range.

## 5. Conclusion

In this study, 80 patients who underwent CCTA examination and FFR examination in the hospital were selected as the research objects. Taking the FFR value of 0.8 as the dividing line, they were divided into the ischemic group (FFR ≤ 0.8) and nonischemic group (FFR > 0.8). The basic data and imaging characteristics of the patients were analyzed. The results showed that CT-FFR based on computer-aided diagnosis system had high accuracy in evaluating myocardial ischemia caused by coronary artery stenosis, and calcification did not affect the diagnostic accuracy of CT-FFR within a certain calcification score range. However, this study is a small sample, single center, and retrospective data, especially CT-FFR-related research, which is lack of large-scale, multicenter, and prospective clinical data to verify. In the future, such studies will be carried out to verify the robustness of its diagnostic efficacy based on larger sample size. Therefore, this study provides a data reference for the clinical accurate diagnosis of cardiovascular diseases.

## Figures and Tables

**Figure 1:** Process of coronary artery automatic segmentation algorithm.

**Figure 2:** CAD System for coronary artery.

**Figure 3:** Function demonstration of coronary artery CAD system module.

**Figure 4:** Normal coronary artery signs ((a) is diastolic; (b) is systolic).

**Figure 5:** Calcification of coronary arteries without stenosis ((a) is CCTA image; (b) is the reconstruction of surface; (c) is corresponding angiography).

**Figure 6:** Calcification of coronary arteries with stenosis ((a) is CCTA image; (b) is the reconstruction of surface; (c) is corresponding angiography).

**Figure 7:** Comparison of the degree of lumen stenosis and characteristic indexes of vulnerable plaque between the two groups ((a) is MDS % and MAS %; (b) is NRS, RI, and EI). Note: ^∗^ indicates that the difference is statistically significant compared with the ischemia group (*P* < 0.05).

**Figure 8:** Quantitative indexes of plaque volume and burden in two groups ((a) is TPV and TPB; (b) is CPV and CPB; (c) is NCPV and NCPB; (d) is LPV and LPB; (e) is FPV and FPB). Note: ^∗^ indicates that the difference is statistically significant compared with the ischemia group (*P* < 0.05).

**Figure 9:** Diagnostic performance of quantitative indexes (MDS %, MAS %, LPV, and LPB) in coronary myocardial ischemia. Note: (a) refers to sensitivity, specificity, and accuracy. (b) is the cut-off value and AUC area.

**Figure 10:** Diagnostic performance of quantitative indexes (TPB, CPV, CPB, TPV) in coronary myocardial ischemia. Note: (a) refers to sensitivity, specificity, and accuracy. (b) is the cut-off value and AUC area.

**Table 1:** Comparison of basic data of patients.

Basic information	Ischemic group	Nonischemic group	*P* value
Age (years old)	54.08 ± 10.11	50.89 ± 7.92	0.632
Male (%)	66.38	63.92	0.583
Height (cm)	161.41 ± 23.58	169.05 ± 21.44	0.591
Weight (kg)	63.94 ± 9.25	68.36 ± 8.11	0.792
Hyperlipemia (%)	27.21	25.66	0.498
Hypertension (%)	62.07	69.44	0.511
Diabetes (%)	25.76	29.51	0.722
Smoker (%)	26.09	30.75	0.537
LDLC (mmol/L)	2.35 ± 0.74	2.48 ± 0.59	0.589
HDLC (mmol/L)	1.24 ± 0.35	1.09 ± 0.21	0.865
TC (mmol/L)	4.25 ± 0.84	4.11 ± 1.05	0.846
FPG (mmol/L)	5.83 ± 1.38	6.13 ± 1.41	0.745
TG (mmol/L)	1.63 ± 0.36	1.44 ± 0.39	0.724

**Table 2:** Diagnostic performance of CT-FFR in two groups of patients.

Index	Ischemic group	Nonischemic group	*P* value
Sensitivity (%)	89.93	93.75	0.673
Specificity (%)	92.07	90.88	0.735
Accuracy rate (%)	95.84	96.24	0.626
Truncated value	60.51	58.22	0.857
AUC area	0.932	0.944	0.776

## Data Availability

The data used to support the findings of this study are available from the corresponding author upon request.
